This article has been retracted.

# Disulfiram Chelated With Copper Inhibits the Growth of Gastric Cancer Cells by Modulating Stress Response and Wnt/β-catenin Signaling

**DOI:** 10.3389/fonc.2020.595718

**Published:** 2020-12-21

**Authors:** Ling Wang, Xiaoke Chai, Run Wan, Hong Zhang, Cong Zhou, Lin Xiang, Maswikiti Ewetse Paul, Yumin Li

**Affiliations:** ^1^ Key Laboratory of Digestive System Tumors of Gansu Province, Lanzhou University Second Hospital, Lanzhou, China; ^2^ Department of Pathology, First Hospital of Lanzhou University, Lanzhou, China; ^3^ Department of Pathology, Lanzhou University Second Hospital, Lanzhou, China

**Keywords:** gastric cancer, disulfiram, copper, apoptosis, autophagy, stress response, Wnt/β-catenin signaling pathway

## Abstract

Disulfiram (DSF) is a well-known drug for alcohol abuse. In recent decades, DSF has been demonstrated to exhibit anti-tumor activity; DSF chelated with copper shows enhanced anti-tumor effect. Our goal was to explore the effect of DSF/Cu complex on the growth and metastasis of gastric cancer (GC) *in vitro* and *in vivo*. DSF/Cu complex suppressed the proliferation, migration of MKN-45 and BGC-823 GC cells. Furthermore, DSF/Cu treatment reduced the tumor volume in GC mouse models with a tumor suppression rate of 48.24%. Additionally, DSF/Cu induced apoptosis *in vitro* in MKN-45 and BGC-823 GC cells in a dose- and time-dependent manner as well as *in vivo* in the xenograft tumor mouse model. Furthermore, DSF/Cu induced autophagy and autophagic flux in MKN-45 and BGC-823 cells, increased the expression of autophagy-related Beclin-1 and LC3 proteins *in vivo*. Additionally, DSF/Cu suppressed aerobic glycolysis and oxidative phosphorylation by reducing oxygen consumption rate and extracellular acidification rate, respectively, in MKN-45 and BGC-823 cells. Treatment with DSF/Cu induced oxidative stress and DNA damage response by elevating the reactive oxygen species levels; increasing the expression of P53, P21, and γ-H2AX proteins; and inhibiting Wnt/β-catenin signaling *in vitro* and *in vivo*. Thus, DSF/Cu suppressed the growth and metastasis of GC cells *via* modulating the stress response and Wnt/β-catenin signaling. Hence, DSF may be used as a potential therapeutic agent for the treatment of GC.

## Introduction

In 2018, gastric cancer (GC) ranked fifth in among all cancers regarding incidence and third regarding cancer-related deaths globally (1). In China, GC occupied the second and third rank in terms of cancer incidences and deaths, respectively, in 2015 (2); however, it was associated with the highest recorded morbidity and mortality in 2013 in Gansu province (3). Although different management techniques and comprehensive therapies have been used for treating GC, their clinical benefits remain unsatisfactory (4). Furthermore, only a few patients with GC are diagnosed at the early stages of the disease. Moreover, metastasis remains the dominating cause of deaths in majority of the cases. In GC patients with metastasis, a 5-year survival rate has been reported to be only 5% (5). Therefore, drugs with high efficacy and low toxicity are required for GC treatment.

Currently, there has been increasing attention in anti-tumor role of the anti-alcoholism drug disulfiram (DSF). Multiple studies have explored the anti-tumor role of DSF in various cancers, such as breast cancer, liver cancer, pancreatic cancer, and so on; moreover, the anti-cancer activity of DSF has been shown to increase when it is chelated with copper (Cu) (6, 7). The underlying mechanisms associated with the anti-cancer activity of DSF may involve inhibition of the proteasome activity, suppression of metastasis, proliferation of cancer stem cell, DNA methylation, and elevation of reactive oxygen species (ROS) as well as the modulation of different signaling pathways (8).

Stress response and genetic aberrations are the universal phenomena associated with tumorigenesis (9). Stress response, including responses to metabolic and oxidative stress, unfolded proteins, heat shock proteins, and DNA damage, plays a dual role in the process of tumor development and progression (10–13). The canonical Wnt/β-catenin signaling pathway is involved in embryonic and organ development and is reportedly activated in GC and plays a pivotal role in the carcinogenesis, invasion, metastasis, progression, and drug resistance of GC cells (14).

The aim of the current study was to explore if DSF chelated with Cu could suppress the growth and metastasis of GC cells using MKN45 GC cell line and tumor xenograft mouse model.

## Materials and Methods

### Chemicals, Reagents, and Instruments

RPMI 1640 medium, fetal bovine serum (FBS), and trypsin-EDTA were purchased from Gibco, USA. Minimum Eagle’s medium (MEM) was obtained from HyClone, USA. Antibiotic/antimycotic solution, kanamycin, puromycin, and dimethyl sulfoxide (DMSO) were obtained from SolarBio, China. DSF was purchased from Selleck, China, whereas CuCl_2_ was obtained from J&K, China. Phenylmethanesulfonyl fluoride (PMSF), radioimmunoprecipitation assay (RIPA) buffer, and bicinchoninic acid (BCA) reagent were obtained from Beyotime, China. Cell counting kit-8 (CCK-8) reagent was purchased from Dojindo, Japan, whereas AnnexinV-FITC (AV-FITC), propidium iodide (PI) and PI kit were purchased from Roche, Germany. Electrochemiluminescence (ECL) was obtained from Biosharp, China. Lipofectamine 2000 (Lip2000) was purchased from Invitrogen, USA, whereas ROS assay kit was obtained from NJJCBIO, China. Seahorse XF Glycolysis Stress Test and XF Cell Mito Stress Test kits were purchased from Agilent, USA. DeadEnd™ Fluorometric TUNEL System was obtained from Promega, USA, whereas antifade mounting medium with DAPI was purchased from SolarBio, China.

### Antibodies

Anti-Bcl 2 (1:2,000; cat. no. 12789-1-AP), anti-Bax (1:2,000; cat. no. 50599-2-LP), anti-Beclin 1 (1:2,000; cat. no. 11306-1-AP), anti-LC3 I/II (1:1,000; cat. no. 14600-1-AP), anti-GAPDH (1:20,000; cat. no. 10494-1-AP), and goat anti-rabbit IgG-HRP (1:10,000; cat. no. SA00001-2) were obtained from Proteintech, China. Anti-P53 (1:1,000; cat. no. 2527S), anti-P21 (1:1,000; cat. no. 2947S), and anti-cyclin D1 (1:1,000; cat. no. 2978S) were purchased from Cell Signaling Technology, USA. Anti-frizzled 7 (1:1,000; cat. no. ab64636), anti-β-catenin (1:2,000; cat. no. ab32572), anti-c-myc (1:5,000; cat. no. ab32072), and anti-γ-H2AX (1:5,000; cat. no. ab2893) were obtained from Abcam, USA. The UltraSensitiveTM SP kit (cat. no. KIT-9710) was purchased from Maixin-Biocompany, China.

### Cell Culture and Transfection

Human gastric carcinoma cell lines of MKN-45, BGC-823 and human embryonic kidney cell line HEK293T were purchased from the Type Culture Collection of the Chinese Academy of Sciences (Shanghai, China). The cells were cultured in RPMI 1640 medium supplemented with 10% FBS at 37°C and 5% CO_2_. Green fluorescent protein-light chain 3 (GFP-LC3) was donated Yunsheng Zhang (Hunan University), and monomeric red fluorescent protein-GFP-LC3 (mRFP-GFP-LC3) plasmid was purchased from Hedgehog Bio (China). MKN-45 and BGC-823 cells were grown overnight in six-well plates (3 × 10^5^ cells per well), and then incubated with a mixture of GFP-LC3 plasmid and Lip2000, which was prepared by using the OptiMEM medium at a ratio of 4μg plasmid/4μl of Lip2000 per well. After 6 h of incubation, the cells were again cultured in RPMI 1640 medium. Following 72 h incubation, the cells were transfected with the lentivirus containing the insert and screened by puromycin. HEK293T cells were cultured overnight in six-well plates (1 × 10^6^ cells per well) and incubated with a mixture of pSPAX2, pMD2G, and mRFP-GFP-LC3 OptiMEM medium.

### Synthesis of Disulfiram/Cu Complex

DSF and CuCl_2_ were dissolved in sterilized water at a molar ratio of 1:1. In the subsequent experiments, the DSF/Cu complex was diluted at required concentrations and used.

### Cell Cytotoxicity Assay

MKN-45 and BGC-823 cells were cultured overnight in 96-well plates (2 × 10^4^ cells per well) followed by treatment with DMSO or varying doses of DSF/Cu (15, 75, 150, 300, or 600 μM) for 12, 24, or 48 h. Then CCK-8 solution (10 μl) was added to the culture, and the cells were further incubated for 2 h. The absorbance was measured at 450 nm by using a microplate reader (Bio-TEK Instruments, USA). The growth inhibition rate was calculated as follows:

Inhibition rate (%)=[(Ac−As)/Ac−Ab]×100,

where As, Ac, and Ab represent the absorbance of treatment, control, and blank groups, respectively.

### Scratch Assay

MKN-45 and BGC-823 cells were cultured in six-well plates (3 × 10^5^ cells per well). When the cells reached a confluence of 90–95%, three scratches per well were performed using a 200 μl pipette tip. Then the cells were treated with DMSO or DSF/Cu (100 or 300 μM) for 24 or 48 h. The migration of the cells was observed by a microscope (Olympus, UK), and the results were analyzed using Image J software.

### Transwell Assay

MKN-45 and BGC-823 cells were treated with DMSO or DSF/Cu (100 or 300 μM) for 24 h. The Transwell chamber was coated with Matrigel (1:9) and placed onto the 24-well plate. The pre-treated cells (1 × 10^5^ cells per well) were suspended in 200 μl of RPMI 1640 medium. The cell suspension and RPMI 1640 medium containing 10% FBS were placed in the apical and basolateral chambers, respectively. Then the cells in the upper chamber were washed away, and the migrated cells were fixed with 4% paraformaldehyde and stained with crystal violet, and images were captured using the light microscope (Olympus, UK).

### Colony Formation Assay

MKN-45 and BGC-823 cells were treated with DMSO or DSF/Cu (100 or 300 μM) for 24 or 48 h. Then GC cells were cultured in 35 mm cell-culture dishes (1,000 cells per well), and the cells were cultured for 1 week. Then the cells were fixed with 4% paraformaldehyde and stained with crystal violet. The number of colonies was analyzed by using Image J software.

### Apoptosis, Reactive Oxygen Species Level, and Autophagy Detection Assays

MKN-45 and BGC-823 cells were cultured overnight in six-well plates (3 × 10^5^ cells per well) and then treated with DMSO or DSF/Cu (100 or 300 μM) for 24 or 48 h. The apoptotic rate of the treated cells was estimated using AV-FITC/PI staining and flow cytometry, and the results were analyzed using FlowJo software (Treestar, USA). The intracellular ROS level was measured using 2′,7′-dichlorodihydrofluorescein diacetate staining and flow cytometry, and the stained cells were observed using a fluorescence microscope. For the estimation of autophagy, MKN-45 and BGC-823 cells with transient GFP-LC3 expression were treated with DMSO or DSF/Cu (100 or 300 μM) for 24 or 48 h, and the green fluorescent intensity was detected by flow cytometry.

### Western Blotting

MKN-45 and BGC-823 cells were cultured overnight in six-well plates (3 × 10^5^ cells per well) followed by treatment with DMSO or DSF/Cu (100 or 300 μM) for 24 or 48 h. The cells were then lysed using a mixture of RIPA buffer and PMSF (1,000:1) followed by protein purification. The protein content in the cell lysate was quantified using BCA assay. The protein samples (20 μg) were separated by 10% or 12% sodium dodecyl sulfate-polyacrylamide gel electrophoresis, transferred to nitrocellulose membrane, and blocked with 5% BSA for 2 h at 37°C. The membranes were subsequently incubated with primary antibodies overnight at 4°C followed by incubation with secondary antibodies for 1 h at room temperature. Finally, the membranes were incubated with ECL and the images were captured with VersaDoc imaging system (Bio-Rad, USA).

### Transmission Electron Microscopy

MKN-45 and BGC-823 cells were obtained after DSF/Cu (100 or 300 μM) treatment for 48 h, fixed in 2.5% glutaraldehyde, dehydrated through a graded series of ethanol solution (50, 70, 80, 90, and 95%), and embedded in resin. The specimens were then cut into ultra-thin sections, stained, and examined under HT7700 transmission electron microscope (HITACHI, Japan).

### Confocal Microscopy

MKN-45 and BGC-823 cells transiently expressing GFP-LC3 and stably expressing mRFP-GFP-LC3 were treated with DMSO or DSF/Cu for 48 h and were imaged using laser scanning confocal microscopy (Carl Zeiss, China).

### Glycolysis and Oxidative Phosphorylation Measurement Assay

MKN-45 and BGC-823 cells (2 × 10^4^ cells per well) were cultured overnight in 24-well plates (Agilent, USA), and then treated with DMSO or DSF/Cu (100 or 300 μM) for 24 or 48 h. To determine the rate of glycolysis and oxidative phosphorylation, oxygen consumption rate (OCR) and extracellular acidification rate (ECAR) were measured using Seahorse XF24 Extracellular Flux Analyzer (Agilent, USA) according to the manufacturer’s instructions.

### Animal Studies

All the mouse experiments were approved by the Ethics Committee of Lanzhou University Second Hospital Animal Center. Male BALB/c nude mice (age: 5–6 weeks, weight: 18–20 g) were purchased from Charles River Laboratories, Inc. Beijing, China. MKN45 cells and Matrigel were mixed at a ratio of 1:1 and the cell suspension was subcutaneously injected into the left upper limbs of the mice. When the tumor reached a volume of approximately 80–100 mm^3^, the mice were randomly assigned into control and DSF/Cu groups (n = 8). The mice were then treated with DMSO (control) or DSF/Cu (5 mg/kg) by oral gavage for 2 weeks. The tumor volume and body weight of the animals was measured every alternate day till the end of the experiment. The tumor volume was calculated as follows: V = 0.5 × L × W^2^, where L and W represent the length and width of the tumor, respectively. The anti-tumor efficacy of DSF/Cu was measured as tumor suppression rate (TSR), which was calculated as follows: TSR (%) = (Vc − Vt)/Vc × 100, where Vc and Vt indicate the tumor volume in the control and treatment group, respectively. At the end of experiment, the mice were sacrificed, tumor tissues were fixed, paraffin embedded, and cut into small tissue sections, which were then used for hematoxylin-eosin (H&E) staining, TUNEL assay, and immunohistochemistry (IHC) analysis. For H&E staining, the slides were deparaffinized, hydrated, stained, and sealed, whereas for IHC staining, the slides were deparaffinized, and rehydrated followed by incubation with the primary and subsequently secondary antibodies. The slides were then stained with 3,3’-diaminobenzidine, counterstained with hematoxylin and analyzed under light microscope (AMG, USA). For TUNEL assay, the slides were deparaffinized, digested with Proteinase K, incubated with DeadEnd™ Fluorometric TUNEL System, mounted in antifade mounting medium with DAPI, and imaged by confocal microscopy.

### Statistical Analysis

Data were analyzed by the Image J and GraphPad Prism 7 software. The differences between two groups were calculated by one-way analysis of variance, and results with P value of <0.05 were considered statistically significant.

## Results

### Disulfiram/Cu Inhibited Viability and Proliferation of Gastric Cancer Cells

As shown in **Figure 1**, DSF/Cu treatment (15–600 µM for 12, 24, or 48 h) inhibited the proliferation of MKN-45 and BGC-823 cells in a dose- and time-dependent manner.

**Figure 1:** DSF/Cu inhibits the viability of GC cells as measured by the CCK-8 assay. **(A, B)** MKN-45 and BGC-823 GC cells were incubated with different doses of DSF/Cu (15, 75, 150, 300 and 600 μM) for 12, 24, or 48 h to assess the cell proliferation inhibition rate. The line graph represents the mean ± SD, n ≥ 3.

### Disulfiram/Cu Inhibited Migration of Gastric Cancer cells

DSF/Cu treatment inhibited the migration of MKN-45 and BGC-823 cells compared to DMSO treatment. As shown in **Figure 2**, the migration rate of treated cells decreased with increasing concentration of DSF/Cu (100–300 μM) and longer period of treatment (24–48 h).

**Figure 2:** DSF/Cu inhibits the migration of GC cells. **(A, C)** MKN-45 and BGC-823 cells were incubated with DMSO or DSF/Cu (100 or 300 mM) for 24 or 48 h, and migration of cancer cells was assessed by scratch assay. Typical scratch assay images and quantifications are shown. **(B, D)** The column chart shows mean ± SD, n ≥ 3. *P < 0.05, ***P < 0.001, and ****P < 0.0001.

### Disulfiram/Cu Inhibited Invasion of Gastric Cancer Cells

As shown in **Figure 3**, the invasion rate was shown to be lower in cells treated with higher concentration of DSF/Cu (300 *vs* 100 μM). Similarly, the migration rate of treated cells decreased with increasing concentration of DSF/Cu (100–300 μM) and longer period of treatment (24–48 h).

**Figure 3:** DSF/Cu inhibits the invasion of GC cells. **(A)** MKN-45 and BGC-823 cells were incubated with DMSO or DSF/Cu (100 or 300 μM) for 24 or 48 h, and cell invasion was assessed by Transwell assay. Representative Transwell images and quantifications are shown. **(B)** The column chart shows mean ± SD, n ≥ 3. ****P < 0.0001.

### Disulfiram/Cu Inhibited Colony Forming of Gastric Cancer cells

MKN-45 and BGC-823 cells treated with DSF/Cu had lower colony forming ability compared to control cells (**Figure 4**). The colony forming ability of the cancer cells reduced drastically with higher concentration of DSF/Cu (300 μM) at 24 or 48 h of treatment.

**Figure 4:** DSF/Cu inhibits the colony forming ability of the GC cells. **(A, C)** MKN-45 and BGC-823 cells were incubated with DMSO or DSF/Cu (100 or 300 μM) for 24 or 48 h, and colony formation assay was performed. Typical colony images and quantifications are presented. **(B, D)** The column chart shows mean ± SD, n ≥ 3. ***P < 0.001 and ****P < 0.0001.

### Disulfiram/Cu Induced Apoptosis in Gastric Cancer Cells

As shown in **Figure 5**, the percentage of apoptotic cells in the control, 100 μM DSF/Cu-treated, and 300 μM DSF/Cu-treated groups was 2.7 ± 0.23%, 8.69 ± 0.38%, and 23.83 ± 2.32%, respectively, after 24 h of treatment. The apoptosis rate further increased to 15.47 ± 0.61% and 42.11 ± 1.29% at concentrations of 100 and 300 μM, respectively, after 48 h of treatment. Furthermore, the expression of B-cell lymphoma-2 (Bcl-2) decreased and that of Bax protein increased in the DSF/Cu-treated cells compared with that in the DMSO (control)-treated cells (**Figure 5**).

**Figure 5:** DSF/Cu treatment induces apoptosis of the GC cells. **(A, B)** Flow cytometry analysis indicates increased rate of apoptosis in MKN-45 and BGC-823 cells treated with DSF/Cu (100 or 300 μM) for 24 or 48 h than that in cells treated with control (DMSO) in a time- and dose-dependent manner. **(C, D)** Western blot analysis indicating decreased Bcl-2 and increased Bax expression in DSF/Cu-treated (100 or 300 μM for 24 or 48 h) MKN-45 and BGC-823 GC cells than that in the DMSO (control)-treated cells in a time- and dose-dependent manner. The column chart shows mean ± SD, n ≥ 3. *P < 0.05, **P < 0.01, ***P < 0.001 and, ****P < 0.0001.

### Disulfiram/Cu Induces Autophagy and Autophagic Flux in Gastric Cancer Cells

The effect of DSF/Cu treatment on autophagy was demonstrated by various methods in MKN-45 and BGC-823 cells (**Figures 6**–**8**). The formation of double-membrane autolysosomes and autophagosomes was observed in DSF/Cu-treated MKN45 cells by transmission electron microscopy (**Figures 6A, B**). Furthermore, western blotting results showed an increase in Beclin1 levels and LC3 II/I ratio in DSF/Cu-treated MKN-45 and BGC-823 cells in a dose and time-dependent manner (**Figures 6C, D**). Additionally, we investigated the distribution of GFP-LC3 in MKN-45 and BGC-823 cells transiently expressing GFP-LC3 (**Figure 7**). The results showed an increase in the distribution of GFP-LC3 in DSF/Cu-treated MKN-45 and BGC-823 cells in a dose and time-dependent manner (**Figure 7A**). This was further confirmed quantitatively by flow cytometry assays (**Figures 7B, C**). The autophagic flux was detected by stably expressing mRFP-GFP-LC3 in MKN-45 and BGC-823 cells. The variation in red and yellow puncta represented a change in autophagic flux. As shown in **Figure 8**, an increase in yellow dots, representing autophagosomes was observed in DSF/Cu-treated MKN-45 and BGC-823 cells compared to that in the control-treated cells, demonstrating a significant induction in autophagic flux in the treated cells.

**Figure 6:** DSF/Cu induces autophagy in GC cells. **(A, B)** Formation of autophagosomes and autolysosomes in DSF/Cu-treated MKN-45 and BGC-823 GC cells was observed by transmission electron microscopy. Red arrowhead indicates autophagosome/autolysosome. **(C, D)** Western blot analysis indicating increased expression of Beclin1 and LC3II/I ratio in MKN-45 and BGC-823 GC cells treated with DSF/Cu (100 or 300 μM) for 24 or 48 h. *P < 0.05, **P < 0.01, ***P < 0.001, and ****P < 0.0001.

**Figure 7:** DSF/Cu increases the expression of GFP-LC3 in GC cells. **(A)** Confocal microscopy, enhanced expression of GFP-LC3 in MKN-45 and BGC-823 GC cells treated with DSF/Cu (100 or 300 μM) for 24 or 48 h. **(B, C)** Increased fluorescence intensity of GFP-LC3 in MKN-45 and BGC-823 cells treated with DSF/Cu (100 or 300 μM) for 24 or 48 h, as shown by flow cytometry analysis. The column chart shows mean ± SD, n ≥ 3. **P < 0.01, ***P < 0.001, and ****P < 0.0001.

**Figure 8:** DSF/Cu treatment (100 or 300 μM for 48 h) induces autophagic flux in MKN-45 and BGC-823 GC cells. **(A)** MKN-45 and BGC-823 cells stably expressing mRFP-GFP-LC3 were constructed. **(B, C)** Confocal microscopy images of autophagosome (yellow puncta) and autolysosome (red puncta) and quantification of yellow (RFP+GFP+) puncta are shown. Magnification, ×600. **P < 0.01 and ****P < 0.0001.

### Disulfiram/Cu Modulates the Stress Response in Gastric Cancer Cells

The role of DSF/Cu on modulating the stress responses was demonstrated by various experimental strategies in MKN-45 and BGC-823 cells. As shown in **Figure 9**, various parameters of OCR, including glycolysis, glycolytic capacity, and glycolytic reserve, were found to be decreased by DSF/Cu treatment, indicating a decrease in the aerobic glycolysis in DSF/Cu-treated MKN-45 and BGC-823 cells. Furthermore, various parameters of ECAR, including basal respiration, maximal respiration, and ATP production, were found to be reduced in DSF/Cu-treated MKN-45 and BGC-823 cells, indicating a reduction in oxidative phosphorylation (OXPHOS). The fluorescence microscopy and flow cytometry results showed that DSF/Cu elevated ROS levels in MKN-45 and BGC-823 cells in a concentration- and time-dependent manner (**Figure 10**). Furthermore, the expression of P53, P21, and γ-H2AX proteins increased in DSF/Cu-treated MKN-45 and BGC-823 cells compared with that in the control cells, with expression being higher at higher concentration (300 *vs* 100 μM) of DSF/Cu (**Figure 11**).

**Figure 9:** DSF/Cu modulates cell metabolism in GC cells. DSF/Cu suppresses aerobic glycolysis and oxidative phosphorylation in MKN-45 cells **(A, C, E, G)** and BGC-823 cells **(B, D, F, H)** treated with DSF/Cu (100 or 300 μM) for 24 or 48 h, as analyzed by Seahorse XF24 analyzer. **(A–D)** DSF/Cu suppresses the aerobic glycolysis by decreasing oxygen consumption rate. **(E–H)** DSF/Cu suppresses oxidative phosphorylation by decreasing extracellular acidification rate.

**Figure 10:** Increase in the ROS levels in GC cells treated with DSF/Cu (100 or 300 μM) for 24 or 48 h. **(A, B)** Increased ROS levels in MKN-45 and BGC-823 GC cells treated with DSF/Cu (100 or 300 μM) for 24 or 48 h, as indicated by enhanced fluorescence intensity. **(C, D)** Increased fluorescence intensity of ROS in MKN-45 and BGC-823 cells treated with DSF/Cu (100 or 300 μM) for 24 or 48 h, as shown by flow cytometry analysis. The column chart shows mean ± SD, n ≥ 3. ***P < 0.001 and ****P < 0.0001.

**Figure 11:** DSF/Cu modulates oxidative stress in GC cells. **(A, B)** Western blot analysis indicating increased expression of oxidative stress associated proteins, P21, P53, and γ-H2AX in DSF/Cu-treated MKN-45 and BGC-823 GC cells. The column chart shows mean ± SD, n ≥ 3. *P < 0.05, **P < 0.01, ***P < 0.001, and ****P < 0.0001.

### Disulfiram/Cu Inhibits Wnt/β-catenin Signaling in Gastric Cancer Cells

As shown in **Figure 12**, DSF/Cu treatment reduced the expression of Wnt/β-catenin signaling pathway related proteins, such as frizzled-7 (Fzd7), β-catenin, C-myc, and Cyclin D1, compared with control treatment. A slight decrease in the expression of these proteins was observed at a concentration of 100 μM of DSF/Cu; however, the decrease was found to be significantly higher at a higher dose of DSF/Cu (300 μM).

**Figure 12:** DSF/Cu treatment modulates Wnt/β-catenin signaling pathway in GC cells. **(A, B)** Western blot analysis indicating decreased expression of Fzd7, β-catenin, C-myc, and Cyclin D1 proteins in MKN-45 and BGC-823 GC cells treated with DSF/Cu (100 or 300 μM) for 24 or 48 h. The column chart shows mean ± SD, n ≥ 3. *P < 0.05, **P < 0.01, ***P < 0.001, and ****P <0.0001.

### Anti-Cancer Activities of DSF/Cu *In Vivo*

The *in vivo* activity of DSF/Cu was demonstrated using a subcutaneous tumor xenograft mouse model of MKN-45 cells. The DSF/Cu (5 mg/kg) group showed a reduction in the tumor volume, as indicated by a TSR of 48.24% (**Figures 13A, B**). As shown in **Figure 13C**, there was no significant difference observed in the body weight between the control and DSF/Cu-treated mice (P = 0.66). Furthermore, H&E staining demonstrated the induction of necrosis was increased by DSF/Cu treatment (**Figure 14A**). The expression of Ki-67 protein, a marker for cellular proliferation, significantly decreased (**Figure 14B**) by DSF/Cu treatment. TUNEL assay demonstrated the induction of apoptosis in the tumor tissues of DSF/Cu-treated mice compared to that in the tissues of DMSO-treated mice (**Figure 15A**). Furthermore, the expression of Beclin1 and LC3 (**Figures 15B, C**). In addition, the oxidative stress associated proteins (P53 and γ-H2AX), and the Wnt/β-catenin signaling associated proteins, including Fzd7, β-catenin, C-myc, and Cyclin D1 were shown to be reduced by DSF/Cu treatment (**Figure 16**).

**Figure 13:** DSF/Cu suppresses the growth of gastric tumors *in vivo*. Tumor xenograft mouse models were treated with DMSO or DSF/Cu (5 mg/kg) by oral gavage every alternate day for 2 weeks and effect of the treatment on various tumor characteristics was assessed by different methods. **(A, B)** DSF/Cu treatment reduces tumor volume compared with control treatment. **(C)** No significant difference in the body weight of the mice between DSF/Cu-treated group and control group was observed. The column chart shows mean ± SD, n ≥ 3. ****P <0.0001.

**Figure 14:** DSF/Cu represses proliferation *in vivo*. **(A)** DSF/Cu treatment induces necrosis in the tumor tissues as shown by H&E staining. **(B)** Immunohistochemistry analysis indicated a decrease in the expression of Ki-67 in the tumor tissues of DSF/Cu-treated mice. The column chart shows mean ± SD, n ≥ 3. ****P < 0.0001.

**Figure 15:** DSF/Cu promotes apoptosis and autophagy in the tumor tissues. **(A)** DSF/Cu promotes apoptosis as assessed by TUNEL assay. **(B, C)** DSF/Cu increases the expression of Beclin1 and LC3 in tumor tissues of DSF/Cu-treated mice, as assessed by immunohistochemistry. The column chart shows mean ± SD, n ≥ 3. ****P < 0.0001.

**Figure 16:** DSF/Cu inhibits DNA damage and Wnt/β-catenin signaling pathway in gastric cancer subcutaneous graft. DSF/Cu increases the expression of P53, γ-H2AX, decreases the expression of Fzd7, β-catenin, C-myc, and Cyclin D1 in the tumor tissues of DSF/Cu-treated mice, as assessed by immunohistochemistry. Representative images of immunohistochemical analysis are presented. The column chart shows mean ± SD, n ≥ 3. *P < 0.05, **P < 0.01, and ***P < 0.001.

## Discussion

Since 1800s, DSF has been used in rubber production (15). Since the year 1940, it has been used for treating alcoholism and currently has been approved by the U.S. Food and Drug Administration (16). Furthermore, the anti-cancer activity of DSF has been explored since 1977 (17). DSF is rapidly converted to diethyldithiocarbamate in the system, which forms a stable complex with Cu; the complex exhibits a stronger anti-tumor effect than DSF alone (18). DSF/Cu complex has been reported to suppress the growth and metastasis of non-small-cell lung cancer (NSCLC), hepatocellular carcinoma, and oral squamous cell carcinoma (6, 19, 20). Zhang et al. found that disulfiram repressed the viability and progression of gastric cancer cells, and inhibited the expression of Wnt/β-catenin by ELISA (21). Therefore, we aimed at exploring the anti-cancer activity of DSF/Cu complex using MKN-45 and BGC-823 GC cells. The cell viability assay showed that DSF/Cu at a concentration of 100 and 300 μM inhibited 50% of the MKN-45 and BGC-823 cells after 12, 24, or 48 h of treatment. Hence, we considered 100 and 300 μM of DSF/Cu for further investigations.

In the current study, DSF/Cu not only inhibited the proliferation but also inhibited the migration and invasion of MKN-45 and BGC-823 cells, indicating its role in the suppression of growth and metastasis of GC cells.

PCD, the cell-intrinsic suicidal pathway, is associated with the development, homeostasis, and pathogenesis of cells (22). Apoptosis is a form of type I PCD (22). Bcl-2 family proteins are important in cell apoptosis and regulate the mitochondrial outer membrane permeabilization (MOMP) (23). The accumulation of BAX–BAK oligomers promote MOMP and results in the release of intermembrane proteins to the cytosol, which leads to apoptosis body formation (24). Our study revealed that DSF/Cu treatment increased the rate of apoptosis in GC cells as well as induced apoptosis *in vivo*, which is agreement with the findings from a previous cancer study (7).

Autophagy (also known as macroautophagy), a form of type II PCD, results in the sequestration of cytoplasmic components, protein aggregates, and organelles and formation of autophagosomes (25, 26). Because of the various cancer types and cancer stages, the dual role of autophagy in cancer development has been reported (27). Beclin1, a homolog of yeast autophagy associated gene-6 (ATG6), regulates the formation of autophagosomes by regulating Bcl-2 family of proteins, ATG14L, ultraviolet radiation resistance-associated gene, vacuolar protein sorting 34 (VPS34), and kinase activity (27–29). Existing studies on GC report varying levels of Beclin1. For instance, increased levels of Beclin1 has been reported to increase autophagy, which may be related to tumorigenesis in GC (30). However, in the poorly differentiated GC cells (MKN-45 and BGC-823 cells) and human GC tissues, the expression of Beclin1 was found to be reduced (31). Our results found that the level of Beclin1 increased after the treatment of MKN-45 and BGC-823 cells with DSF/Cu, which is in accordance with the finding from a study that showed BECN1 to be a haploid-insufficient tumor suppressor in carcinoma (32). LC3, a homolog of yeast ATG8, contains LC3-I and LC3-II chains. Cytosolic LC3-I is activated by ATG7, which is then transferred to ATG3 and results in the formation of the membrane-bound protein form, LC3-II (33). LC3-II is involved in the formation and expansion of autophagosomes, and thus autophagy (34). In our study, expression of Beclin1 and LC3-II/I ratio were found to be increased in MKN-45 and BGC-823 cells and in xenograft tumor tissues after DSF/Cu treatment. Furthermore, green/red fluorescent protein-tagged-LC3 (GFP/RFP-LC3) has been widely used to monitor the role of LC3 in the formation of autophagosomes and the dynamic changes associated with them, *in vitro* and *in vivo* (35). In the current study, we successfully constructed MKN-45 and BGC-823 cells transiently expressing GFP-LC3, and confirmed that DSF/Cu treatment increases the accumulation of punctate GFP-LC3. In addition, we showed that LC3-II specifically localizes to autophagosomes and is degraded in the autolysosome. The autophagic flux may be analyzed by mRFP-GFP-tagged LC3 (35). Similar to that in the lysosomal lumen, GFP is degraded under acidic conditions, whereas mRFP is stable under this condition. Thus, an mRFP signal indicates the formation of autolysosomes, whereas yellow puncta (coexistence of GFP and RFP fluorescence) represents a phagophore or an autophagosome (35). In the current study, we constructed MKN-45 and BGC-823 cells stably expressing mRFP-GFP-LC3 and showed increased accumulation of yellow LC3-II puncta in DSF/Cu-treated cells, indicating increased autophagic flux, which is consistent with the findings reported for non-small cell lung cancer (36). Thus, our findings suggest that DSF/Cu treatment induces apoptosis and autophagy in MKN-45 and BGC-823 GC cells, leading to cell death.

Redox homeostasis is important in maintaining the cellular functions and cell survival. ROS triggers oxidative stress, which plays a pivotal role in the development and treatment of tumors (37). However, the role of ROS in cancer progression is controversial. ROS at low and moderate levels is associated with tumor formation, whereas it is responsible for severe cellular damage and cell death at higher levels (37). In the current study, a drastic increase in ROS levels was observed in DSF/Cu-treated MKN-45 and BGC-823 cells. Similar to our findings, multiple studies have demonstrated the role of DSF/Cu in elevating ROS levels in different cancers, such as head and neck squamous cell carcinoma, NSCLC, and oral squamous cell carcinoma (38–40). Exogenous and endogenous stressors have been reported to induce DNA damage (41), which are repaired by DNA damage response (DDR) mechanisms, thus restoring the genome integrity (42). The DDR mechanisms include ATR signaling, double-strand break repair (DSB), homologous recombination repair, non-homologous end joining repair, mismatch repair, base excision repair (BER), and nucleotide excision repair (NER) (42). As a tumor suppressor gene and cyclin-dependent kinase inhibitor, respectively, P53 and P21 play a role in cell cycle, apoptosis, DDR, and immune response (43–46). P53 mediates DDR signaling by regulating the transcription of downstream genes, whereas P21 mediates DDR by increasing the rate of BER, DSB, and NER (47, 48). In the current study, DSF/Cu treatment elevated the expression P53 and P21 in MKN-45 and BGC-823 cells. These findings were agreement with the results reported in nasopharyngeal cancer cells, where the expression of both P53 and P21 were shown to increase after DSF/Cu treatment (49). Furthermore, γ-H2AX, a marker for DSB, is associated with the mediator of DNA damage checkpoint 1 (MDC1) (50, 51). We showed an increase in γ-H2AX in MKN-45 and BGC-823 cells treated with DSF/Cu, similar to the findings from studies on prostate cancer and atypical teratoid/rhabdoid tumors (52, 53). Thus, our findings suggested that DSF/Cu triggered oxidative stress and DDR by increasing ROS, P53, and P21 levels.

The Warburg effect, according to which cancer cells undergo aerobic glycolysis rather than OXPHOS even in the presence of oxygen, is a well-known phenomenon in cancer growth and proliferation (54). Further, metabolic reprogramming is important during cancer metastasis (55). Wnt/β-catenin signaling has been known to increase the glucose uptake and repress mitochondrial respiration (52). For instance, Wnt signaling reduces aerobic glycolysis in colon cancer (56), whereas mitochondrial function is suppressed *via* C-myc, the downstream gene of Wnt/β-catenin signaling, in triple-negative breast cancer (57). In prostatic cancer, DSF/Cu regulates cell metabolism (52), whereas in glioblastoma, DSF suppresses the Wnt signaling pathway (58). Our study showed that DSF/Cu not only inhibited glycolysis and OXPHOS by repressing OCR and ECAR in MKN-45 and BGC-823 cells but also decreased the levels of Fzd7, β-catenin, C-myc, and Cyclin D1 in MKN-45 and BGC-823 cells, indicating the deregulation of Wnt/β-catenin signaling pathway in GC.

In the tumor xenograft mouse model, DSF/Cu inhibited tumor volume, as indicated by a TSR of 48.47%. Further, no change in the body weight between DSF/Cu-treated and control mice groups indicated the safety and low toxicity of DSF/Cu. Additionally, DSF/Cu inhibited cancer cell proliferation, induced necrosis, apoptosis, and autophagy *in vivo*. Moreover, DSF/Cu treatment triggered oxidative stress and modulated the expression of proteins associated Wnt/β-catenin signaling in the tumor tissues.

As this study was originally designed to explore the role of DSF/Cu in inhibiting the growth of GC cells, a positive control was not used; this is a limitation of the current study. Multiple studies have demonstrated that DSF-nanoparticles have enhanced anti-cancer effect (18). In the future, we plan to perform nano-modification of DSF and use docetaxel as a positive control to further explore the role of DSF in cancer. Furthermore, we are hopeful that more preclinical trials will be conducted before DSF is used in clinical practice.

In conclusion, our study demonstrated that DSF/Cu exhibits anti-cancer effects by modulating stress responses and the Wnt/β-catenin signaling pathway in MKN-45 and BGC-823 GC cells and xenograft tumor mouse model. Therefore, DSF may be a beneficial chemotherapeutic agent for the treatment of GC.

## Data Availability Statement

The original contributions presented in the study are included in the article/supplementary materials; further inquiries can be directed to the corresponding author.

## Ethics Statement

The animal study was reviewed and approved by the Ethics Committee of Lanzhou University Second Hospital Animal Center.

## Author Contributions

LW designed and performed the experiments as well as prepared and edited the original manuscript draft. XC designed the experiments. RW, HZ, CZ, and LX conducted the experiments. MP edited and reviewed the manuscript. YL supervised the complete project and edited the manuscript. All authors contributed to the article and approved the submitted version.

## Funding

Our work was financially supported by the grants from National Natural Science Foundation of China (grant no. 31770537) and International Science and Technology Cooperation Project of Gansu Province (grant no. 18YF1WA113).

## Conflict of Interest

The authors declare that the research was conducted in the absence of any commercial or financial relationships that could be construed as a potential conflict of interest.

## Abbreviations

DSF, disulfiram; GC, gastric cancer; ROS, reactive oxygen species; PCD, programmed cell death; FBS, fetal bovine serum; MEM, minimum Eagle’s medium; DMSO, dimethyl sulfoxide; PMSF, phenylmethanesulfonyl fluoride; RIPA, radioimmunoprecipitation assay; BCA, bicinchoninic acid; ECL, electrochemiluminescence; Cu, copper; OCR, oxygen consumption rate; ECAR, extracellular acidification rate; TSR, tumor suppression rate; H&E, hematoxylin-eosin; IHC, immunohistochemistry; OXPHOS, oxidative phosphorylation; NSCLC, non-small-cell lung cancer; MOMP, mitochondrial outer membrane permeabilization; DDR, DNA damage response; DSB, double-strand break repair; BER, base excision repair; NER, nucleotide excision repair.
